The article "Online and Offline Interaction Model of International Chinese Education Based on Few-Shot Learning" was retracted in 2023. Reasons: unreliable results or conclusions; concerns about the data; concerns about the peer review; concerns about the citations.

# Online and Offline Interaction Model of International Chinese Education Based on Few-Shot Learning

**DOI:** 10.1155/2022/8281670

**Published:** 2022-05-05

**Authors:** Fei Cao, Jing Cai

**Affiliations:** ^1^School of Humanities, Hangzhou Normal University, Hangzhou 311121, China; ^2^Rotterdam Business School, Rotterdam University, University of Applied Science, Kralingse Zoom 91 3063, ND Rotterdam, Netherlands

## Abstract

Few-shot learning is a method to acquire learning ability in a small amount of sample data scenarios. This paper aims to study an online and offline interaction model applied to international Chinese education and teaching based on the few-shot learning method. It first expounds an overview of international Chinese education, including the connotation and characteristics of the hybrid mode of online teaching and offline teaching in international Chinese education, then designs an online and offline interactive model, and finally compares it with a baseline model and a traditional single teaching model. The experimental data shows that the accuracy and recall rate of the international Chinese education online and offline interaction model based on few-shot learning both reach 70%, which verifies its effectiveness.

## 1. Introduction

Language is not only one of the important media for the transmission of culture, but also an indispensable part of the expression of human thoughts and ideas. With the diversified development of world culture and the rapid increase of China's economic and technological strength, Chinese has become another popular language after English. The charm and connotation of Chinese are more and more appreciated and valued by many countries. According to research data released by the Ministry of Education, more than 70 countries around the world have incorporated Chinese language education into their educational systems and structures. The number of people studying Chinese overseas has also exceeded 20 million, and the number of overseas Chinese education institutions is also increasing every year, as shown in Figure 1. International Chinese education has entered a period of vigorous development. However, with the outbreak of the new crown epidemic, traditional offline education has been hit. International Chinese education has transformed from offline to online development. However, due to the particularity of Chinese teaching, and because online education is still in the early stage of exploration, there are still many limitations in the current international Chinese education. For example, online classroom learning is full of difficulties, low flexibility, and the interactive experience between students and teachers, which has brought many negative effects [1].

The article "Online and Offline Interaction Model of International Chinese Education Based on Few-Shot Learning" was retracted in 2023. Reasons: unreliable results or conclusions; concerns about the data; concerns about the peer review; concerns about the citations.

The Chinese interpretation of few-shot learning is small sample learning. As the name implies, it is to master the ability of learning and generalization in a small number of samples. Learning in this way can enable humans to obtain an initial target set for learning in a very small number of individual categories. Humans can not only learn object permanence through this target set, but also generalize and apply it to other objects based on this target set. This type of method often plays its own role in task scenarios where data or supervision information is difficult to obtain. It can not only find suitable models for scarce sample tasks, but also assist in data- and computing-intensive data collection, such as image retrieval, object tracking and language modeling, and one-shot architecture search.

Many academics have studied the subject of more-shot training in recent years. Shi Y proposed a self-determination training-based multishot modeling algorithm. The algorithm has a large number of resources and a simple network design. Finally, simulation results show that this algorithm can improve model recognition by 5% to 10%. Chen M proposed a novel diversity transfer network generation framework to address the lack of diversity in few-shot learning. He also confirmed that the generation framework has state-of-the-art results in the few-shot learning method based on feature generation [2] through experimental results. Lv Q proposes the new more-shot learning method in conjunction with programming observation and replaces the mean square error loss function with L1Loss and BCEloss. The test's final results show that the method has an average accuracy of 97.25 percent in the data set, indicating that it is effective [3]. In manipulated microbot systems, Zhang D proposed a data-driven approach to stability and depth analysis. It also demonstrates the method's generality by adapting to microrobots of various shapes using a multishot learning curve [4]. Aharchaou M gives an example of machine learning in action. This example is based on recent advancements in deep learning systems, as well as Siamese networks' few-shot learning capability, which has been shown to generalize well to new datasets [5]. Deng S used meta-learning and unsupervised language models to solve the problem of negating common language features implicit across tasks in few-shot tasks and confirmed that pretraining is a promising solution in many few-shot tasks [6]. Few-shot learning was proposed by Wang Y to address the problem of machine learning being hindered in applications with small datasets. He also looks into the setting, technical, applied, and theoretical aspects of the few-shot learning problem in order to give researchers ideas for future research [7]. Silver T proposes a powerful but general prior and a learning algorithm that, when combined, can learn interesting policies from few shots and shows that this method is a good fit for tasks with sparse training data [8]. In the field of civil aviation emergency management, Hong W proposed a few-shot learning method. Finally, experiments show that the method can solve the problem of automatic updating of concepts and relationships in large-scale domain ontologies while also providing good data support, and using few-shot machine learning [9–11] to train general neural network models in cell lines also has many advantages for high-throughput screening of individual patients. To summarize, many scholars have studied the few-shot learning method and application in depth after several years of research. However, there are few studies that integrate it with the international Chinese education model of online and offline interaction, and previous studies still have some flaws, as shown in Table 1.

The article "Online and Offline Interaction Model of International Chinese Education Based on Few-Shot Learning" was retracted in 2023. Reasons: unreliable results or conclusions; concerns about the data; concerns about the peer review; concerns about the citations.

Therefore, this paper incorporates the few-shot learning method to establish an online and offline interaction model in order to further promote the long-term development of international Chinese education. It also investigates the current state of international education and teaching, as well as problems and practical teaching strategies. It proposes a novel educational interaction research direction that can effectively improve the quality of Chinese education and teaching, offer suggestions for improvement and improvement for international Chinese communication, and generate new ideas for Chinese education and teaching research.

## 2. International Chinese Education Based on Few-Shot Learning

### 2.1. Overview of International Chinese Education

On the basis of the first Chinese international education, international Chinese education is being developed. It is primarily written in the form of a second language for foreigners and foreign Canadians who do not speak English as their first language. Although international Chinese education and teaching have an offline component, traditional offline education cannot be adapted in the face of the new epidemic. Traditional education should keep up with the times, build digital and networking, and develop online teaching and learning, as shown in Figure 2, in order to promote the healthy and sustainable development of international Chinese education. Of course, this does not imply that international education and teaching in Canada will replace traditional schooling, nor that offline education will become the predominant teaching method. Modern technology and techniques will not completely replace traditional face-to-face instruction, but they are more likely to introduce a variety of teaching positions in various combinations and sizes. It is believed that it will be able to fully benefit from Chinese online education and that online education can be used as an aid and complement to offline education if the level of international online education in Canada is raised and the quality of education is improved.

The article "Online and Offline Interaction Model of International Chinese Education Based on Few-Shot Learning" was retracted in 2023. Reasons: unreliable results or conclusions; concerns about the data; concerns about the peer review; concerns about the citations.

#### 2.1.1. The Connotation of the Mixed Mode of Online Teaching and Offline Teaching

The hybrid teaching mode that combines online and offline is an organic combination of online teaching and traditional face-to-face classroom teaching, which integrates multiple elements (teacher, student, classroom, environment, etc.). It is through the transformation of modern information technology means and teaching methods. On the basis of conforming to the laws of language communication, the complementarity between online learning and offline classroom teaching can be realized, so as to achieve the best learning effect. Pure online teaching or offline teaching can no longer fully meet the current Chinese learning needs. Compared with traditional face-to-face classroom teaching and fully online teaching, the online-offline hybrid teaching mode has a deeper meaning. This teaching model neither unilaterally emphasizes the dominant position of students and ignores the dominant position of teachers, nor unilaterally emphasizes online teaching and ignores the emotional communication between teachers and students in traditional face-to-face classrooms. The blended teaching combining online and offline may become a normalized teaching mode in the postepidemic era.

#### 2.1.2. Characteristics of the Hybrid Mode of Online Teaching and Offline Teaching

*(1) Multichannel Teaching*. At present, the online and offline teaching modes of international Chinese education and teaching are still not closely connected, and the two have not been organically combined. The hybrid teaching mode that combines online and offline teaching cannot simply separate the two, and online Chinese teaching can not only be used as an auxiliary to offline teaching, but must be a necessary teaching link. The offline Chinese teaching in the blended teaching should not just copy the teaching activities in the traditional face-to-face classroom teaching, but should further develop the teaching activities based on the previous results of online Chinese teaching.

*(2) Complete Teaching Links*. The first stage of the learner's learning process is mainly information transmission, and the second stage is mainly the absorption and internalization of the teaching content. The blended teaching mode of Chinese online teaching optimizes the classroom structure and promotes the rationalization of teaching content distribution. The flipped classroom teaching mode adopts the teaching form of “learning knowledge before class—consolidation and practice in class”, and learners can conduct autonomous learning of target knowledge by watching videos online. Practical language practice is carried out in the offline classroom, and the target knowledge is applied in practice.

*(3) Targeted Teaching*. The online Chinese teaching in the online and offline hybrid teaching can make up for the lack of offline classroom teaching time to a certain extent. However, due to the lack of deep participation of teachers, the effect of learners will be difficult to guarantee; teachers should pay attention to the design of teaching content and target language environment in offline Chinese classroom teaching. By recording the learner's Chinese learning situation, the teacher supervises the learner's learning progress, which is helpful for the teacher to better grasp the teaching progress of the offline classroom and make the teaching activities more targeted.

*(4) Interactive Teaching*. Training Canada online and offline can not only affect the quality of teachers, but also reflect the high position of students. Teachers teach relevant target knowledge online and complete information transfer; offline practice is a specific exercise of language points. By strengthening the interaction between teachers and students in the classroom, learners can complete the absorption and internalization of knowledge, so that online teaching can better serve offline teaching. At the same time, offline education can be better adapted to online education, in order to achieve a positive attitude and improve the quality of teaching and learning.

The article "Online and Offline Interaction Model of International Chinese Education Based on Few-Shot Learning" was retracted in 2023. Reasons: unreliable results or conclusions; concerns about the data; concerns about the peer review; concerns about the citations.

### 2.2. Design of Online and Offline Interactive Model Based on Few-Shot Learning

Few-shot learning is used in this paper to identify the features of intent classification and semantic understanding in international Chinese education, and the two models are combined with algorithms to create a complete online and offline interaction model. The sample input model of the support set and query set must first be encoded, and the data must then be converted into a sample semantic vector that contains semantic information and is more conducive to model learning for the task of intent classification. The class vector of each class in the support set is then obtained by extracting some intentional category features from the semantic vector of the support set sample. Finally, they calculate the loss function and finish the backpropagation by comparing the class vector with the query set sample semantic vector. The few-shot intent recognition model is divided into three parts based on these three basic steps, as shown in Figure 3: encoding module, induction module, and relation module.

The main task of the encoding module is to receive the sample input of support set and query set and encode them into sample semantic vectors. In this study, a bidirectional long-term and short-term memory network with self-attention mechanism was used to form the encoder. Given a set of input text *x*=(*x*_1_, *x*_2_,…, *x*_*T*_) represented by a sequence of word embedding, use *Bi* − LSTM to process this set of text:

(1) $$\begin{array}{c} \overset{⟶}{h_{t}}=\overset{⟶}{\text{LSTM}}\left(x_{t},h_{t-1}\right),\\ \overset{\leftarrow }{h_{t}}=\overset{\leftarrow }{\text{LSTM}}\left(x_{t},h_{t+1}\right). \end{array}$$

Connect $\overset{⟶}{h_{t}}$ and $\overset{\leftarrow }{h_{t}}$ to obtain a hidden state *h*_*t*_, and record all *T* hidden states as *H*=(*h*_1_, *h*_2_,…, *h*_*T*_). The length of each text sample is different, and we need to encode it as a fixed-size embedding, which can be achieved by choosing a linear combination of *T* latent vectors LSTM in *H* [12]. Computing the linear combination requires a self-attention mechanism that takes the entire hidden state *H* of LSTM as input and outputs a weight to a:

(2) $$\begin{array}{c} a=\text{soft }\max\left(W_{a2}\tanh\left(W_{a1}H^{T}\right)\right). \end{array}$$

The definitions of all parameters in (2) are shown in Table 2.

From this, the semantic vector *e* of an input sample is finally expressed as the weighted sum of *H* for the self-attention weight *a*:

(3) $$\begin{array}{c} e=\sum_{t=1}^{T}a_{t}\cdot h_{t}. \end{array}$$

The sample semantic vector of all samples in the support set and query set can be obtained through the encoding module. Among them, the sample semantic vector *e*^*s*^ of the support set needs to be input into the induction module, while the sample semantic vector *e*^*q*^ of the query set is directly input to the relation module [13]. The induction module needs to summarize some essential characteristics of the intent category according to the *K* samples of each class in the support set, that is, according to the sample semantic vector of the support set, abstract a class vector *c* of each class, so this part is called the induction module:

(4) $$\begin{array}{c} {\left\{e_{ij}^{s}\in R^{2u}\right\}}_{i=1,\ldots ,C,\;j=1,\;K}↔{\left\{C_{i}\in R^{2u}\right\}}_{i=1,\ldots ,C}. \end{array}$$

In previous studies, there have been some computational methods, for example, directly adding the semantic vectors of each sample, or taking the average value of the semantic vectors of the samples as a class vector to obtain abstract class vectors. But in few-shot learning, because the number of samples is too small, it is not enough to cover a wider and general situation. This kind of simple algorithm will bring great chance, and the noise brought by each sample is huge, and the capsule network can solve this problem very well [14]. The capsule network adopts an idea of inverse rendering, which can predict the overall features of the high-level from the local features of the bottom layer, so that the model has better generalization, as shown in Figure 4.

The article "Online and Offline Interaction Model of International Chinese Education Based on Few-Shot Learning" was retracted in 2023. Reasons: unreliable results or conclusions; concerns about the data; concerns about the peer review; concerns about the citations.

In the task of intent classification, the sample semantic vector can be regarded as a local feature, while the class vector that needs to be abstracted can be regarded as the overall feature. Through the dynamic routing algorithm, the coupling coefficient between the sample vector and the same kind of vector is increased, and the coupling coefficient with other class vectors is reduced, so as to obtain a class vector that can dynamically change according to the sample vector and has better generalization. According to the dynamic routing algorithm, it is first necessary to multiply the sample vector by a transformation matrix to obtain the prediction vector:

(5) $$\begin{array}{c} {\hat{e}}_{ij}^{s}=W_{s}e_{ij}^{s}. \end{array}$$

Here is a slight change to the original dynamic routing algorithm: In order to be able to support sets of various sizes (that is, *C* and *K* can take any value), let all sample semantic vectors in the support set share a transformation matrix *W*_*s*_ ∈ *R*^2*u*×2*u*^, instead of setting a *W*_*ij*_ for each sample. This transformation matrix *W*_*s*_ can encode important spatial and other relations between low-level features (sample semantics) and high-level features (intent categories), and it is also learned to update through backpropagation.

Next, the coupling coefficient *d* needs to be learned, which is used to represent the probability that each sample semantic vector is routed to each class. And the size of *d* will be automatically corrected in multiple iterations of the dynamic routing algorithm, and the sum of the coupling coefficients for each class of sample vectors is guaranteed to always be 1 by the softmax function:

(6) $$\begin{array}{c} d_{i}=\text{soft }\max\left(b_{i}\right), \end{array}$$

where *b*_*i*_ is the logarithm of the coupling coefficient, initialized to 0 in the first iteration.

A weighted sum is performed on all the predicted vectors obtained in each class, so that the predicted class vector is obtained:

(7) $$\begin{array}{c} {\hat{c}}_{i}=\sum_{j}d_{ij}\cdot {\hat{e}}_{ij}^{s}. \end{array}$$

The modulus of ${\hat{c}}_{i}$ represents the probability of the existence of the class it represents, so the nonlinear function squash is used in the capsule network to replace the activation function relu in the traditional neural network, as shown in Figure 5.

The article "Online and Offline Interaction Model of International Chinese Education Based on Few-Shot Learning" was retracted in 2023. Reasons: unreliable results or conclusions; concerns about the data; concerns about the peer review; concerns about the citations.

It is ensured that short vectors can be compressed to lengths close to 0 and long vectors to lengths close to 1, and the direction of the vectors remains unchanged [15].

(8) $$\begin{array}{c} \text{squash}\left(x\right)=\frac{{\left|\left|x\right|\right|}^{2}}{1+{\left|\left|x\right|\right|}^{2}}\frac{x}{\left|\left|x\right|\right|}. \end{array}$$

Finally get the class vector *c*_*i*_:

(9) $$\begin{array}{c} c_{i}=\text{squash}\left({\hat{c}}_{i}\right). \end{array}$$

The final step of each iteration of the dynamic routing algorithm is to update the logarithm of the coupling coefficient of *b*. If the dot product of *c*_*i*_ and *b*_*ij*_ is large, there is a top-down feedback, which increases the coupling coefficient of this sample and decreases the coupling coefficient of other samples. Each *b*_*ij*_ is updated by

(10) $$\begin{array}{c} b_{ij}=b_{ij}+{\hat{e}}_{ij}^{s}\cdot c_{i}. \end{array}$$

To sum up, the entire algorithm process is shown in Table 3, where *r* is a hyperparameter representing the number of iterations of the algorithm. The algorithm finally outputs a class vector *c*_*i*_ for each class.

The relation module measures the correlation between each sample semantic vector *e*_*i*_^*q*^ in the query set and each class vector *c*_*j*_ output by the induction module, and it outputs a scalar between 0 and 1 to represent this correlation score. The calculation formula of the scoring function is as follows:

(11) $$\begin{array}{c} r_{ij}=\text{sigmoid}\left(\text{SIM}\left(e_{i}^{q},c_{j}\right)\right). \end{array}$$

Among them, SIM is a similarity function, which can choose cosine similarity, dot product similarity, and so on. Cosine similarity measures the similarity of two vectors by calculating the cosine value of the angle between the two vectors and pays more attention to the similarity in direction, while the dot product similarity directly calculates the dot product of the two vectors, which can directly measure the similarity of the length and direction of the two vectors. The higher the similarity of two vectors, the larger their dot product. Moreover, compared with the calculation steps of cosine similarity, dot product similarity is simpler to implement, and it is the simplest similarity measurement method, which can improve the efficiency of the model. For the above two reasons, this paper uses the dot product similarity to calculate the similarity of two vectors, namely:

(12) $$\begin{array}{c} \text{SIM}\left(e_{i}^{q},c_{j}\right)=e_{i}^{q},c_{j}. \end{array}$$

In this paper, the mean square error (MSE) is used as the loss function. For matching query set samples (*x*_*q*_, *y*_*q*_) and intent categories, the closer the correlation score *r*_*iq*_ is to 1, the better it will be, while for unmatched samples and categories, the closer *r*_*iq*_ to 0, the better. In episode, for the input support set *S*_support_ and query set *S*_quiry_, the loss function of *C* classes is defined as

(13) $$\begin{array}{c} L\left(S_{\text{support}},S_{\text{quiry}}\right)=\sum_{j=1}^{C}\sum_{i=1}^{n}{\left(r_{ij}-1\cdot \left(y_{i}==j\right)\right)}^{2}. \end{array}$$

The loss function is derived and backpropagated, and all parameters in the above three modules are updated until the best parameters are learned.

The article "Online and Offline Interaction Model of International Chinese Education Based on Few-Shot Learning" was retracted in 2023. Reasons: unreliable results or conclusions; concerns about the data; concerns about the peer review; concerns about the citations.

The few-shot semantic understanding joint model is improved on the basis of the structure of the few-shot intent recognition model. The overall structure is also divided into three parts: cocoding module, separate induction module, and fusion scoring module.  Figure 6 is the basic structure of the joint model of few-shot semantic understanding.

The coencoding module is one of them, and it is used to coencode the input model's support and query set samples not only to get the sample semantic vector, but also to get the sample sequence vector for the semantic slot filling task. The class vectors for the intent and semantic slots are inducted separately using a separate induction module. The fusion scoring module scores the intent and semantic slot matching based on the similarity between the sample vector and the class vector, but the semantic slot scoring is not done separately, but rather combines the results of the intent classification, so that the sample intent category provides some support for semantic slot annotation. Finally, the backpropagation loss is reduced by combining the loss functions of the two tasks. The coencoding module's primary function is to receive support and query set sample input. For semantic slot prediction and intent classification, they are encoded to produce a sample sequence vector and a sample semantic vector for each sample. The sample semantic vector is an attention-based vector obtained by weighting and calculating the sample sequence vector, which can better focus on the important information in the sample, and the sample sequence vector incorporates the context information of the entire sample during the encoding process.

Given a set of input text *x*=(*x*_1_, *x*_2_,…, *x*_*T*_) represented by a sequence of word embedding, first process this set of text using *Bi* − LSTM:

(14) $$\begin{array}{c} \overset{⟶}{h_{t}}=\overset{⟶}{\text{LSTM}}\left(x_{t},h_{t-1}\right),\\ \overset{\leftarrow }{h_{t}}=\overset{\leftarrow }{\text{LSTM}}\left(x_{t},h_{t+1}\right). \end{array}$$

Connect $\overset{⟶}{h_{t}}$ and $\overset{\leftarrow }{h_{t}}$ to obtain a hidden state *h*_*t*_, and record all *T* hidden states as *H*=(*h*_1_, *h*_2_,…, *h*_*T*_). Among them, each *h*_*T*_ is a word vector representation that obtains the information before and after the current word, and *H* is used as the sample sequence vector *e*^*s*^ of this input sample, namely:

(15) $$\begin{array}{c} e^{s}=H=\left(h_{1},h_{2},\ldots ,h_{T}\right). \end{array}$$

The attention calculation is performed on *H*, and the calculation method is the same as that of the few-shot intent recognition model, and the sample semantic vector *e*^*I*^ of each sample is obtained:

(16) $$\begin{array}{c} e^{I}=\sum_{t=1}^{T}a_{t}\cdot h_{t}. \end{array}$$

Finally, the sample sequence vector *e*^*S*_*S*_^ and the sample semantic vector *e*^*S*_*I*_^ of each sample of the support set and the sample sequence vector *e*^*Q*_*S*_^ and the sample semantic vector *e*^*Q*_*I*_^ of each sample of the query set are output to the common coding module.

The article "Online and Offline Interaction Model of International Chinese Education Based on Few-Shot Learning" was retracted in 2023. Reasons: unreliable results or conclusions; concerns about the data; concerns about the peer review; concerns about the citations.

Input *e*^*S*_*I*_^ and *e*^*S*_*S*_^ of the support set samples output by the coencoding module into the induction module, which are used to calculate the class prototype representation *c*^*I*^ for each intent category and the semantic slot label class vector *c*^*S*^ for each semantic slot label category:

(17) $$\begin{array}{c} {\left\{e_{i}^{S_{I}}\in R^{2u}\right\}}_{i=1,\ldots ,s}⟶{\left\{c_{j}^{I}\in R^{2u}\right\}}_{j=1,\ldots ,C_{I}},\\ {\left\{e_{i}^{S_{S}}\in R^{2u}\right\}}_{i=1,\ldots ,s}⟶{\left\{c_{j}^{S}\in R^{2u}\right\}}_{j=1,\ldots ,C_{S}}. \end{array}$$

Among them, the class prototype vector is still obtained by the dynamic routing algorithm, and the semantic slot label class vector is obtained by TapNet.

## 3. Online and Offline Interactive Model Test

This paper evaluates and tests the online and offline interaction model of international Chinese education based on few-shot learning. Then it is used in teaching practice to verify the validity of the model from the aspects of teaching quality and learning effect, students' experience, and acceptance.

### 3.1. Evaluation Test

The online and offline interactive model evaluation test of international Chinese education based on few-shot learning uses the FewJoint dataset as the experimental dataset. The parameters it uses in the process of building the model and training the model are shown in Table 4

The performance evaluation index of the interactive model adopts the internationally common PRF evaluation index, namely, the precision rate (Precision, P), the recall rate (Recall, R) and the F value. In order to verify the effect of the model, this experiment uses the prototype network as the baseline model and conducts training tests in the six fields of idiomsDic, drama, timesTable, length, story, and constellation of the dataset, and the test results are shown in Figures 7 and 8.

The article "Online and Offline Interaction Model of International Chinese Education Based on Few-Shot Learning" was retracted in 2023. Reasons: unreliable results or conclusions; concerns about the data; concerns about the peer review; concerns about the citations.

Figure 7(a) shows the accuracy test results of the model proposed in this paper.

Figure 7(b) shows the accuracy test results of the prototype network model.

It can be seen from Figure 7 that the model proposed in this paper has an overall training accuracy of 71.31% in the six fields of the dataset: idiomsDic, drama, timesTable, length, story, and constellation; the training accuracy of the prototype network in the six fields of idiomsDic, drama, timesTable, length, story, and constellation of the dataset is 60.03%.

Figure 8(a) shows the recall test results of the model proposed in this paper.

Figure 8(b) shows the recall test results of the prototype network model.

It can be seen from Figure 8 that the model proposed in this paper has an overall training recall rate of 70.15% in the six fields of idiomsDic, drama, timesTable, length, story, and constellation of the dataset; the recall rate of the prototype network training in the six domains of idiomsDic, drama, timesTable, length, story, and constellation of the dataset is 57.99%.

### 3.2. Teaching Practice

This experiment takes foreign students majoring in international Chinese education in a university as the experimental object, with a sample size of 50 people, who are divided into two classes. Class A adopts the online and offline interactive teaching mode proposed in this paper for Chinese learning, and class B adopts a single online mode for Chinese learning. The students of the two classes have basically the same level of Chinese proficiency and related theoretical knowledge and are at the same starting point. Through a semester of teaching practice, the test data of the teaching quality and learning effect, students' experience, and acceptance of the four key stages of teaching were compared and analyzed. The analysis results are shown in Figures 9 and 10.

Figure 9(a) shows the test of teaching quality and learning effect under the online and offline interactive teaching mode.

Figure 9(b) shows the test of teaching quality and learning effect under a single online teaching mode.

It can be seen from Figure 9 that, under the online and offline interactive teaching mode, the overall average of the teaching quality of the four key teaching stages reached 86.28 points, and the overall average of the learning effect reached 82.85 points; under the single online teaching mode, the overall mean of teaching quality in the four key stages of teaching is 78.65 points, and the overall mean of learning effect is 73.68 points.

The article "Online and Offline Interaction Model of International Chinese Education Based on Few-Shot Learning" was retracted in 2023. Reasons: unreliable results or conclusions; concerns about the data; concerns about the peer review; concerns about the citations.

Figure 10(a) is the test of students' experience and acceptance under the online and offline interactive teaching mode.

Figure 10(b) is a test of students' experience and acceptance under a single online teaching mode.

As can be seen from Figure 10, under the online and offline interactive teaching mode, the overall average score of students' experience in the four key stages of teaching reached 86.23 points, and the overall average score of students' acceptance reached 90.38 points; under the single online teaching mode, the overall average score of students' experience in the four key stages of teaching is 80.75 points, and the overall average score of students' acceptance is 76.70 points.

## 4. Discussion

Through the evaluation test data of the online and offline interaction model based on few-shot learning and the prototype network baseline model, the following conclusions can be drawn:

1. In terms of the accuracy of the model, the overall mean of the online and offline interactive model based on few-shot learning in the training and testing of the dataset is 11.28% higher than the overall mean of the prototype network baseline model in the training and testing of the dataset, which shows that the online-offline interaction model based on few-shot learning has superior accuracy.
2. At the model recall level, the overall mean of the online and offline interaction model based on few-shot learning in the training and testing of the dataset is 12.16% higher than the overall mean of the prototype network baseline model in the training and testing of the dataset, which shows that the online-offline interactive model based on few-shot learning is also superior in retrieval performance.
3. Through the teaching practice data of the online and offline interactive teaching mode based on few-shot learning and the traditional single online teaching mode, the teaching quality and learning effect, students' experience, and acceptance, the following conclusions can be drawn.
4. In terms of teaching quality and learning effect, the overall mean of teaching quality under the online and offline interactive model teaching mode based on few-shot learning is 7.63 points higher than the overall mean of teaching quality under the single online teaching mode; the overall mean of the learning effect is 9.17 points higher than the overall mean of the learning effect under the single online teaching mode.
5. In terms of student experience and acceptance, the overall mean of students' experience under the online and offline interactive model teaching mode based on few-shot learning is 5.48 points higher than the overall mean of students' experience under the single online teaching mode; the overall mean of student acceptance is 13.68 points higher than the overall mean of student acceptance under the single online teaching mode; and the overall mean of student acceptance is 13.68 points higher than the overall mean of student acceptance under the single online teaching mode.

The article "Online and Offline Interaction Model of International Chinese Education Based on Few-Shot Learning" was retracted in 2023. Reasons: unreliable results or conclusions; concerns about the data; concerns about the peer review; concerns about the citations.

The entire comparative experimental data shows that when all other experimental conditions are held constant, the online and offline interactive model test data based on few-shot learning performs better in terms of model accuracy and teaching practice results after model scoring and teaching practice test. It demonstrates that the few-shot learning-based online and offline interaction model can improve the level and quality of international Chinese education and teaching, thereby promoting the development of international Chinese education.

## 5. Conclusion

The continuous updating and development of information technology have promoted the modernization of international Chinese education. A new round of Chinese teaching has begun to change, and online and offline Chinese teaching will become an important development direction for international Chinese education. The combination of few-shot learning method and international Chinese education and teaching is beneficial not only to its own diversified development, but also to international Chinese education to solve the teaching restrictions caused by the epidemic and improve the level of intelligent teaching.

There are still many deficiencies in the research of this paper. The depth and breadth of the research in this paper are not enough, without taking into account some interfering factors involved in the teaching practice process, and the evaluation of the teaching mode is also restricted by many factors. And our academic level research is also limited; the research on the online and offline interaction model of few-shot is still in the preliminary stage. In the future work, the model performance will be improved from more angles based on the existing technology and level, and the teaching methods of international Chinese education will be continuously optimized.

## Figures and Tables

**Figure 1:** Growth and changes of overseas Chinese education institutions.

**Figure 2:** Online and offline teaching of international Chinese education.

The article "Online and Offline Interaction Model of International Chinese Education Based on Few-Shot Learning" was retracted in 2023. Reasons: unreliable results or conclusions; concerns about the data; concerns about the peer review; concerns about the citations.

**Figure 3:** Few-shot intent recognition model structure.

**Figure 4:** Capsule network structure diagram.

**Figure 5:** Activation function distribution map.

**Figure 6:** Few-shot semantically understands the basic structure of the federated model.

**Figure 7:** Model accuracy evaluation test.

**Figure 8:** Model recall evaluation test.

**Figure 9:** Teaching quality and learning effectiveness test.

**Figure 10:** Student experience and acceptance test.

**Table 1:** Weaknesses of previous studies.

Sequence	Insufficiency	Influence
1	More qualitative discussions, less quantitative research	Not objective enough
2	More micro research, less macro research	Not comprehensive enough
3	More experience summaries, less theoretical discussions	Not deep enough

**Table 2:** Definition of formula parameters.

Sequence	Parameter	Paraphrase
1	*W*_*a*1_ ∈ *R*^*d*_*a*_×2*u*^	Weight matrix
2	*W*_*a*2_ ∈ *R*^*d*_*a*_^	Weight matrix
3	*d*_*a*_	Hyperparameters
4	*u*	The size of the hidden state vector for each one-way LSTM

**Table 3:** Algorithmic process.

Dynamic routing algorithms in induction modules		
Sequence of steps	1:	For all samplesk *j*=1,…, *K*, in class *i*:
	2:	*b*_*ij*_=0
	3:	${\hat{e}}_{ij}^{s}=W_{s}{\hat{e}}_{ij}^{s}$
	4:	for *r* : iterations do
	5:	*d*_*i*_=softmax(*b*_*i*_)
	6:	${\hat{c}}_{i}=\sum_{j}d_{ij}\cdot {\hat{e}}_{ij}^{s}$
	7:	$c_{i}=\text{squash}\left({\hat{c}}_{i}\right)$
	8:	For all samples *j*=1,…, *K*, in class *i*:
	9:	$b_{ij}=b_{ij}+{\hat{e}}_{ij}^{s}\cdot c_{i}$
	10:	return *c*_*i*_

**Table 4:** Experimental parameter settings.

Serial number	Parameter name	Parameter value
1	Batch size	4
2	Learning rate	L *e* − 5
3	Balance parameters *α*	0.7

## Data Availability

There is no data availability in statement.
